The article "High-Performance Triboelectric Devices via Dielectric Polarization: A Review" was published in 2021. Journal: Nanoscale Res Lett.

# High-Performance Triboelectric Devices via Dielectric Polarization: A Review

**DOI:** 10.1186/s11671-021-03492-4

**Published:** 2021-02-12

**Authors:** Minsoo P. Kim, Doo-Seung Um, Young-Eun Shin, Hyunhyub Ko

**Affiliations:** 1 School of Energy and Chemical Engineering, Ulsan National Institute of Science and Technology (UNIST), Ulsan, South Korea; 2 Department of Electrical Engineering, Sejong University, Seoul, Republic of Korea

**Keywords:** Dielectric polarization, Triboelectric, Relative permittivity, Energy harvesting, Self-powered sensor

## Abstract

Energy harvesting devices based on the triboelectric effect have attracted great attention because of their higher output performance compared to other nanogenerators, which have been utilized in various wearable applications. Based on the working mechanism, the triboelectric performance is mainly proportional to the surface charge density of the triboelectric materials. Various approaches, such as modification of the surface functional group and dielectric composition of the triboelectric materials, have been employed to enhance the surface charge density, leading to improvements in triboelectric performances. Notably, tuning the dielectric properties of triboelectric materials can significantly increase the surface charge density because the surface charge is proportional to the relative permittivity of the triboelectric material. The relative dielectric constant is modified by dielectric polarization, such as electronic, vibrational (or atomic), orientation (or dipolar), ionic, and interfacial polarization. Therefore, such polarization represents a critical factor toward improving the dielectric constant and consequent triboelectric performance. In this review, we summarize the recent insights on the improvement of triboelectric performance via enhanced dielectric polarization.

## Introduction

Piezoelectric, pyroelectric, and triboelectric devices have attracted great attention as energy harvesting devices for power generation from surrounding environments, such as water, wind, light, temperature, and vibration [1]. In addition to the power sources, these devices can be used as self-powered sensors for varied applications such as electronic skins, healthcare monitoring devices, and robotics [2]. Among them, triboelectric devices display relatively higher output performances when a couple of triboelectric materials are contacted [3–6]. The produced triboelectric signals can be used for directly operating electric devices [7–11] or monitoring the mechanical or chemical stimuli on the devices [4]. The triboelectric devices can be simply designed for the simple fabrication, low cost, excellent output performance, and flexibility when compared with other technologies, which are advantageous for self-powered wearable applications [12].

The article "High-Performance Triboelectric Devices via Dielectric Polarization: A Review" was published in 2021. Journal: Nanoscale Res Lett.

Triboelectricity occurs owing to contact electrification and electrostatic induction between dissimilar triboelectric materials. The mechanical contact induces the compensated opposite charges on each triboelectric layer owing to the contact electrification, and the mechanical separation results in the current flow through the external circuit because of electrostatic induction. Therefore, the triboelectric output performance is directly affected by the surface charges on triboelectric layers.

For high triboelectric output performances, efficient surface charge generation during contact electrification and effective charge transfer during electrostatic induction are necessary. Therefore, it is crucial to select suitable triboelectric contact-pair materials and design optimum device structures. Based on their working mechanism, four different types of triboelectric devices consisting of dielectric materials as triboelectric layers have been reported [5]. There are two categories of triboelectric devices based on the types of triboelectric contact pair materials: dielectric-to-dielectric and conductor-to-dielectric contact mode devices (Fig. 1a) [13]. In the former, two dielectric plates, with thicknesses *d*_*1*_ and *d*_*2*_, as well as relative dielectric constants *ε*_*r,1*_ and *ε*_*r,2*_, respectively, are stacked face to face as triboelectric layers, and the electrode layers are deposited on the outer dielectric surface. The distance (*x*) between the two triboelectric layers is varied under a periodic mechanical force.

**Fig. 1:** Dielectric-based triboelectric device and dielectric polarization: **a** Theoretical models for parallel-plate contact-modes and equivalent circuit diagram for dielectric-to-dielectric and conductor-to-dielectric TENG (Reproduced from Ref. [21]. Copyright 2014 Royal Society of Chemistry). **b** Real (*ε*') and imaginary part (*ε*") of the dielectric constant as a function of frequency in a polymer having interfacial, orientational, ionic, and electronic polarization mechanisms (Reproduced with permission from Ref. [32, 33]. Copyright 2012 American Chemical Society)

Subsequently, the contacted triboelectric layer surfaces have opposite surface charges but the same density (*σ*) through contact electrification. When the triboelectric layers begin to separate from each other owing to the increasing distance, a potential difference (*V*) is induced between the two electrodes by the amounts of transferred positive/negative charges (+*Q*/*–Q*). Similarly, in the conductor-to-dielectric contact mode without the dielectric 1 layer, metal 1 is used as both the top triboelectric layer and the top electrode. In this device structure, there are two parts of charges in metal 1: the triboelectric charges ($S \times \sigma$) and the transferred charges between the two electrodes (*–Q*), thereby leading to ($S\sigma - Q$) of the total charges in metal 1. Considering the contact mode triboelectric devices mentioned above, the output performance can be derived based on electrodynamics as follows [13]:

1 $$V = - \frac{Q}{{S\varepsilon_{0} }}\left( {d_{0} + x\left( t \right)} \right) + \frac{\sigma x\left( t \right)}{{\varepsilon_{0} }}$$

2 $$\begin{aligned}&V_{{{\text{OC}}}} = \frac{\sigma \cdot x\left( t \right)}{{\varepsilon_{0} }},\quad { }I_{{{\text{SC}}}} = \frac{{{\text{d}}Q_{SC} }}{{{\text{d}}t}},\\&{ }Q_{{{\text{SC}}}} = \frac{S\sigma x\left( t \right)}{{d_{0} + x\left( t \right)}},\quad { }d_{0} = \mathop \sum \limits_{i = 1}^{n} \frac{{d_{i} }}{{\varepsilon_{r,i} }}{ }\end{aligned}$$

The effective dielectric thickness *d*_0_ is defined as the summation of all the thicknesses of dielectric *d*_*i*_ divided by its relative permittivity *ε*_*r,i*_. Based on Eq. 2, the triboelectric performance is directly affected by the surface charge density ($\sigma$) of the dielectric layers.

The article "High-Performance Triboelectric Devices via Dielectric Polarization: A Review" was published in 2021. Journal: Nanoscale Res Lett.

Previously, the surface modification of triboelectric materials or the introduction of highly dielectric materials has been reported to increase the surface charge density. Surface modification, such as the control of surface morphology [14–17] or the introduction of charged ions [18–21], increases surface charge density by enlarging the surface area or triboelectric polarity between the triboelectric pair layers. In addition to tuning the surface property, an increase in the dielectric constant can enhance the capacitance of the dielectric layer, thereby resulting in an increase in the surface charge density [6, 22, 23]. In a parallel-plate capacitor model, the surface charge density can be related to the capacitance of the dielectric layer as follows [23–25]:

3 $$\sigma=\frac{CV}S,\quad C=\frac{S\varepsilon\varepsilon_0}d$$

where *C* and *S* indicate the capacitance and contact area, respectively. From Eq. 3, since the capacitance (*C*), which is a factor capable of improving the surface charge density in a dielectric contact mode triboelectric device [6], increases with the dielectric constant and/or the reduction in the thickness of the dielectric layer, the surface charge density is directly proportional to the ratio of the dielectric constant to the thickness (*ε*/*d*). Similarly, in the triboelectric device, the capacitance of the tribo-dielectric layer can be expressed from Eq. 2 as:

4 $$C=\frac{Q_\text{SC}}{V_\text{OC}}=\frac{\varepsilon_0S}{d_0+x\left(t\right)}$$

For instance, using a porous dielectric layer in a triboelectric device is an efficient way to greatly enhance the ε/*d* ratio by simultaneously increasing the dielectric constant and decreasing the thickness when the dielectric layer is pressed under external pressure, thereby significantly enhancing the surface charge density [17, 23, 26, 27] even when the same triboelectric layers are used. Therefore, the dielectric constant of the triboelectric layer is an effective factor to improve the surface charge density better than the surface potential determined by the selection of triboelectric pair materials.

The article "High-Performance Triboelectric Devices via Dielectric Polarization: A Review" was published in 2021. Journal: Nanoscale Res Lett.

Although the dielectric constant of a triboelectric material is an important factor in the enhancement of triboelectric performances, there have been no comprehensive discussions on the principles and strategies to increase the dielectric constant. Previously, several excellent reviews on triboelectric devices, including triboelectric materials and their working mechanisms, had been reported [3–6, 12, 21, 28, 29]; however, only a few studies on dielectric-induced triboelectric devices have been reported to date. Herein, we introduce the basics of dielectric polarization and demonstrate that the output performances of triboelectric devices can be significantly controlled and enhanced by the design of dielectric materials with controlled dielectric polarization.

## Dielectric Polarization for Enhanced Triboelectric Performance

The dielectric constant (or relative permittivity) is defined as a factor whereby the applied electric field is decreased through the dielectric polarization of materials, which can be enhanced by engineering dielectric materials through the introduction of dielectric additives or the modification of chemical structures, thereby leading to various dielectric phenomena. Dielectric polarization can be divided into electronic, vibrational (or atomic), orientational (or dipolar), ionic, and interfacial polarization (Fig. 1b) [30–33]. Electronic and atomic polarizations are induced by the distortion of negative electrons and positive nuclei in an atom in an opposite direction to the external electric field, thereby acquiring electric dipole moments, which occur in the resonance regime above the infrared frequencies (> 100 GHz). As polarization-based materials, such as semiconductors, have no dielectric loss below 1 GHz, they are the most desired for practical applications ranging from a few Hz to 1 GHz. However, most organic polymers exhibit lower dielectric constants (< 10) than semiconducting materials because of the intrinsic nature of their molecular bonding, which cannot induce electronic and atomic polarization. To further induce electronic and atomic polarizations in the polymers, the polymer chain structures should involve larger atoms with polarizable electrons, such as Si, Ge, or Sn, than the basic polymer compositions [34–36]. Although Si-based polymers, such as polysiloxanes or their derivatives, are synthesized, the dielectric constant is no greater than 3–4. Therefore, it is difficult to increase the electronic/atomic polarization in insulating polymers.

The article "High-Performance Triboelectric Devices via Dielectric Polarization: A Review" was published in 2021. Journal: Nanoscale Res Lett.

In polymers, whereas the electronic and atomic polarizations are limited to enhancing the dielectric constant because of the intrinsic molecular bonding structure, the other dipolar, ionic, and interfacial polarizations can be utilized to improve the dielectric constant. Dipolar (orientation) polarization is caused by the reorientation of permanent molecular dipole moments in the polymers or nanocomposites including nanoparticles or dipolar moieties, which is affected by the phase structures (amorphous or crystalline), temperature, and frequency (usually < 10 MHz) [32, 33]. The modification of dipole structures enables the preparation of dipolar glass, ferroelectric, and relaxor ferroelectric polymers [30]. For example, the dipole orientation of polyvinylidene fluoride (PVDF)-derivatives leads to the formation of a *β*-phase, thereby increasing the dielectric constant, which enhances the triboelectric performance [37, 38]. Ionic polarization can be caused by relative displacements between positively and negatively charged ions under an external force [30, 39]. Therefore, polymers with ionic components can be used to enhance the capacitive performance through ionic polarization. For instance, the ionic components (e.g., NaCl and LiCl) in hydrogels are polarized under an external field, leading to the formation of electric double layers, which results in the improvement of triboelectric performance [40–43]. Interfacial polarization is induced by the reorganization of space charges at interfaces in dielectric composites [30, 31]. Therefore, interfacial polarization is observable in all multicomponent dielectric systems, including semi-crystalline polymers, polymer blends, or nanocomposites with high-*k*- or conducting-nanofillers. Recently, polymer nanocomposites with high-*k* nanoparticles, which improve the net dielectric constant, thereby leading to the enhancement of the surface charge density, and thus the triboelectric performance, have been utilized in triboelectric devices [23, 44, 45]. In the following sections, we introduce some examples to demonstrate the enhancement of triboelectric output performance through an increase in the dielectric constant.

The article "High-Performance Triboelectric Devices via Dielectric Polarization: A Review" was published in 2021. Journal: Nanoscale Res Lett.

## Interfacial Polarization in High-Permittivity Nanoparticle/Polymer Composites

High-permittivity nanoparticles are utilized to improve the dielectric constants of polymer nanocomposites owing to the polarization at the interface between the polymer and nanoparticles. Because inorganic (e.g., barium titanate (BaTiO_3_) nanoparticles and nanowires) or conductive (e.g., metal nanoparticles, carbon nanotubes, and graphene) nanomaterials are widely employed in polymer matrices to increase the net dielectric constant, polymer composites with various additives have higher dielectric constants than base polymers, thereby leading to improved triboelectric performances. Chen et al. prepared a sponge-like polydimethylsiloxane (PDMS) film, including high-*k* nanoparticles (SiO_2_, TiO_2_, BaTiO_3_, and SrTiO_3_), to enhance triboelectric performances (Fig. 2a) [23]. Because SrTiO_3_ exhibits higher permittivity than the others, PDMS with SrTiO_3_ displays a higher dielectric constant. This can also be caused by the space charge polarization at the interface between the PDMS and SrTiO_3_ particles. Notably, the triboelectric output performance is improved by the increase in capacitance through the increased *ε*_r_/*d*_PDMS_ during the contact process. In addition to dielectric nanoparticles, different kinds of high-permittivity materials, such as Al-doped BaTiO_3_ and CaCu_3_Ti_4_O_12_, are applied in the triboelectric layers, leading to an improved dielectric constant and the resultant triboelectric performance (Fig. 2b) [44, 45]. On the other hand, the addition of conductive materials enables the formation of micro-capacitor structures in the polymer matrix, which can induce space charge accumulation at the interface between the polymer matrix and additives. This type of interfacial polarization is caused by the larger difference in conductivity between the polymer and conducting additives.

**Fig. 2:** Triboelectric performances enhanced by interfacial polarization in high-permittivity nanoparticle/polymer composites: **a** Dielectric nanoparticle/sponge PDMS composite-based triboelectric nanogenerator (Reproduced with permission from Ref. [23]. Copyright 2016 American Chemical Society). **b** Contact-separation mode triboelectric nanogenerator with P(VDF-TrFE) and PDMS-high dielectric particle composite films as the friction layers (Reproduced from Ref. [45]. Copyright 2018 Royal Society of Chemistry)

Therefore, polymer composites with metal or carbon-based materials exhibit increased dielectric constants compared to pure polymers, leading to the enhancement of surface charge density and the resultant triboelectric performance (Fig. 3) [6, 46]. Although high-permittivity polymer composites are widely used as triboelectric negative materials, there are some limitations regarding improving the output performance: (1) There is an optimized ratio of additives in the polymer matrix because excessive additives cause leakage current [46, 48] or reduced surface friction area [23, 49], thereby resulting in a decrease in output performance. (2) The additives should be homogeneously dispersed in the polymer matrix to improve the interfacial polarization because the aggregated nanoparticles interrupt interfacial polarization through the reduction of the interfacial area between the polymer and nanoparticles.

The article "High-Performance Triboelectric Devices via Dielectric Polarization: A Review" was published in 2021. Journal: Nanoscale Res Lett.

**Fig. 3:** Triboelectric performances enhanced by interfacial polarization in polymer composites with metal or carbon-based materials: **a** GPs@PDMS composite-based triboelectric nanogenerator (Reproduced from Ref. [82]. Copyright 2015 Royal Society of Chemistry). **b** Liquid–metal-inclusion-based triboelectric nanogenerator with sandwiched dielectric stacks (Reproduced from Ref. [48]. Copyright 2019 Royal Society of Chemistry)

## Interfacial Polarization in Multilayer Polymer Films

For random phase nanoparticle/polymer composites, interfacial polarization is difficult to control because precisely controlling the amount and dispersion of nanoparticle is required [30]. In multilayer dielectrics, interfacial polarization can be easily controlled because all the interfaces are perpendicular to the electric field, resulting in uniform space charge accumulation at the multilayer interfaces and enhanced dielectric constant. Multilayer polymer dielectrics have been widely investigated to enhance their dielectric constant via interfacial polarization between dissimilar polymer layers [50]. Interfacial polarization occurs when the space charges (electrons and ions) are accumulated at the interface between two dissimilar materials with large contrasts in permittivity and electrical conductivity under an external field [30]. Kim et al. [51] and Feng et al. [52] demonstrated the effect of bilayer films with a larger difference in the relative permittivity on the triboelectric output performance (Fig. 4a,b). The addition of lower dielectric layers between the conductive layer and electrode causes charge trapping or storage in the dielectric film, thereby leading to an increased charge density. The charge accumulation could be caused by the increased polarization at the interface of bilayer films through the large difference in the permittivity or conductivity between PVDF and insulating films. On the other hand, our group demonstrated the effect of a bilayer film consisting of polymers with different fluorine units and polyethylene terephthalate (PET) insulating layers on the output performance (Fig. 4c) [53]. Notably, fluorinated polymers with three fluorine units in the side chain (poly(2,2,2-trifluoroethyl methacrylate), PTF) are coated on PET substrates with a lower dielectric constant, thereby increasing the dielectric constant, which is caused by the improved interfacial polarization at the interface between the semi-crystalline PTF and PET. Consequently, the PTF–PET exhibited a higher triboelectric performance than the other fluorinated polymer films. Based on the abovementioned results, heterogeneous dielectric multilayer films can be a robust design to enhance the triboelectric performance of flexible or wearable devices.

The article "High-Performance Triboelectric Devices via Dielectric Polarization: A Review" was published in 2021. Journal: Nanoscale Res Lett.

**Fig. 4:** Triboelectric performances enhanced by interfacial polarization in multilayer polymer films: **a** Triboelectric nanogenerator consisting of PVDF/PDMS double layer and Nylon 6/PDMS double layer with various PDMS interlayer thicknesses (Adapted from Ref. [51]. Copyright 2018 Elsevier). **b** Triboelectric nanogenerator without and with PI as transition layer for charge storage (Adapted from Ref. [52]. Copyright 2017 Elsevier). **c** Bilayer triboelectric nanogenerator based on fluorinated polymers with different kinds of fluorine units (Reproduced from Ref. [53]. Copyright 2018 Elsevier)

## Ionic Polarization in Ionic Polymer Gels

In the polymer matrix including the ionic components except impurity ions, ionic polarization promotes the formation of an electric double layer (EDL) at the interface between the polymer electrolyte and the electrode, thereby leading to the enhancement of the dielectric constant [30, 39, 54]. Polarization is often utilized in energy storage devices, such as capacitors (e.g., supercapacitors or EDL capacitors) and batteries [55]. According to the Helmholtz equation, the capacitance can be expressed as *C ≈ kε*_*0*_*/λ*, where *k*, *ε*_*0*_*,* and *λ* are the effective dielectric constant of the EDL, vacuum permittivity, and Debye screening length (or the thickness of the double layer), respectively. In a triboelectric device, ionic components, such as symmetric or asymmetric ion pairs and ionic liquids, in polymeric materials are often employed. Since poly(vinyl alcohol) (PVA) is a type of negative triboelectric material because of the hydroxyl groups in the polymer backbone, it can interact with different types of ion pairs. When an external electric field is applied, ionic polarization can occur owing to the relative displacements between the positive and negative ions, thereby contributing to EDL formation at the interface between the triboelectric layers. Ryu et al. [43] prepared PVA-based solid polymer electrolytes (SPEs) with symmetric or asymmetric ions as positive or negative triboelectric layers, respectively (Fig. 5a). After the contact process with pristine PVA, different surface potentials were systematically measured by the effect of different types of ionic doping. For example, the SPEs become negative or positive triboelectric materials after the addition of phosphoric acid (H_3_PO_4_) with more cations than anions or calcium chloride (CaCl_2_) with more anions than cations, respectively, because the cations or anions create additional electron charged or unoccupied states. Practically, it is shown that an ionic conductor consisting of PVA with borax solution or poly(acylamide) with lithium chloride is applied in biomechanical energy harvesting and tactile sensing applications, which enhances triboelectric performances through the EDL formation (Fig. 5b) [41, 42, 56]. Similarly, Zou et al. [40] fabricated a bionic stretchable nanogenerator consisting of an elastomer Ecoflex and sodium chloride (NaCl) solution inspired by the structure of the ion channels on the cytomembrane of the electrolyte in an electric eel. By combining the effects of triboelectrification through flowing liquid and electrostatic induction through polarized ions, the device harvests mechanical energy from underwater human motion with an open-circuit voltage over 10 V. Furthermore, Lee et al. [56] investigated the triboelectric performance when a nanogenerator was connected to an ion gel unit composed of an ionic liquid and poly(vinylidene fluoride-co-hexafluoropropylene), making a broad and sluggish voltage profile because of the large relaxation time of the polarized ions (Fig. 5c). Ionic gel-based triboelectric devices enable the fabrication of ultrastretchable, transparent, and waterproof wearable devices, although the devices should be encapsulated by the elastomeric matrix to prevent ion leakage.

The article "High-Performance Triboelectric Devices via Dielectric Polarization: A Review" was published in 2021. Journal: Nanoscale Res Lett.

**Fig. 5:** Triboelectric performances enhanced by ionic polarization in an ionic polymer gel: **a** SPE-triboelectric nanogenerator based on PVA with different kinds of ions (Reproduced with permission from Ref. [43]. Copyright 2017 Wiley–VCH). **b** Soft skin-like triboelectric nanogenerator that enables both biomechanical energy harvesting and tactile sensing by hybridizing elastomer and ionic hydrogel (PAAm-LiCl) as the electrification layer and electrode, respectively (Reproduced under the terms of the CC-BY-NC 4.0 license. Ref. [41]. Copyright 2017, The American Association for the Advancement of Science). **c** Triboelectric-ion-gel system, which consists of the triboelectric nanogenerator and the ion gel units (Reproduced from Ref. [56]. Copyright 2018 Elsevier)

## Dipolar Polarization in Ferroelectric PVDF Derivatives

Dipolar (orientational) polarization is another strategy to enhance the dielectric constant with low dielectric loss, which is caused by the increased dipole moment through the aligned dipoles in the phase structures of the polymer chains. Typical examples are PVDF and its derivatives. The polymers have permanent dipole moments since the unidirectional *β*-phase is formed, leading to an increase in the dielectric constant and the resultant triboelectric performance. Cheon et al. [37] demonstrated high-performance triboelectric nanogenerators based on PVDF-silver nanowire (AgNW) composite nanofibers (Fig. 6a). The introduction of AgNWs into PVDF increases the ratio of the *β*-phase to the *α*-phase through the interaction between AgNWs and PVDF molecular chains, thereby resulting in an improved dielectric constant, which enables charge trapping at the PVDF-AgNW dielectric layer. In addition to the metal sources, Seung et al*.* [38] introduced semiconducting nanoparticles (BaTiO_3_) into a ferroelectric copolymer matrix (poly(vinylidenefluoride-trifluoroethylene), PVDF-TrFE) (Fig. 6b). The triboelectric performance is significantly enhanced after the poling process, which is over 150 times larger than that of typical polytetrafluorethylene-based triboelectric nanogenerators. Unlike the heterogeneous polymer composites, our group recently demonstrated the effect of ferroelectric multilayer nanocomposites on triboelectric performance (Fig. 6c) [57]. The multilayered dielectric films consisting of alternating PVDF-TrFE and BaTiO_3_ layers display a higher dielectric constant (17.1) than the pure PVDF-TrFE film (13.9) and single PVDF-TrFE/BaTiO_3_ nanocomposite (15.9) because of the interfacial polarization between the copolymer and nanoparticle layers, as explained in the section on the multilayered dielectric film (Fig. 4). Sequentially, the triboelectric output performance increases compared to the single-layered films. Although ferroelectric polymer nanocomposites improve the triboelectric output performance owing to the increased dielectric constant through the high ferroelectric polarization, there is a limitation in increasing the output performance because of the percolation threshold of the additives.

**Fig. 6:** Triboelectric performances enhanced by dipolar polarization in ferroelectric PVDF composites: **a** Triboelectric nanogenerator based on the PVDF–AgNW composite and nylon nanofibers prepared through electrospinning methods (Reproduced with permission from Ref. [37]. Copyright 2018 Wiley–VCH). **b** Ferroelectric composite-based triboelectric nanogenerator (Reproduced with permission from Ref. [38]. Copyright 2017 Wiley–VCH). **c** Multilayered PVDF-TrFE/BTO-based triboelectric nanogenerator (Reproduced with permission from Ref. [57]. Copyright 2020 American Chemical Society)

On the other hand, the dipole moment can be modified by introducing polar single molecules [58], such as –CN, –NO_2_, and –SO_2_–, or polar polymers [59–61], including polystyrene, poly(2-hydroxyethyl methacrylate), and poly(dopamine methacrylamide), which allow the rotation of dipoles in the free volume of polymers, thereby leading to an improvement in the dielectric constant. Dipolar polarization has been recently utilized to increase the dielectric constant of triboelectric materials by attaching polar groups with large dipole moments to the side chain of polymers [22]; Lee et al. demonstrated that the PVDF-graft copolymer remarkably increased the triboelectric output performance (Fig. 7). Poly(tert-butyl acrylate) (PtBA) with different grafting ratios was introduced into the PVDF chain, leading to enhanced dipole moment by π-bonding and polar ester groups in PtBA, which improved the dielectric constant and subsequently the triboelectric output performance. In addition to the grafting polymer, polymer dielectrics with nanostructured domains increase the dielectric constant by dipolar orientational polarizability [62]. Although polymer-based dielectric materials have some advantages, such as solution processability and flexibility, few studies wherein such a polarization in triboelectric devices is employed have been reported so far.

The article "High-Performance Triboelectric Devices via Dielectric Polarization: A Review" was published in 2021. Journal: Nanoscale Res Lett.

**Fig. 7:** Triboelectric performances enhanced by dipolar polarization in PVDF-graft copolymer: PVDF-grafting polymer-based triboelectric nanogenerator. **a** Dipole moments of bare PVDF and PVDF-*g*-PtBA and **b** their dielectric properties and triboelectric performances (Reproduced under the terms of the CC-BY-NC 4.0 license. Ref. [22]. Copyright 2017, The American Association for the Advancement of Science)

## Conclusions and Outlooks

Self-powered wearable and implantable electronic devices are essential, especially since the development of Internet-of-Things (IoT) technology. Since the triboelectric effect is one of the most frequently experienced phenomena in everyday life, triboelectric devices are a promising energy harvester for self-powered wearable devices combined with other types of applications. In the development of the IoT industry, electronic devices require miniaturization and multifunctionality, which need high output performances. Although triboelectric devices with high output performances have been developed by employing device structures with combined working modes [63–65], it is necessary to enhance the output performance for multiple devices.

The article "High-Performance Triboelectric Devices via Dielectric Polarization: A Review" was published in 2021. Journal: Nanoscale Res Lett.

Until now, research has been focused on the development of triboelectric pair materials (usually negative triboelectric materials), whereas dielectric tribo-materials have rarely been investigated. As dielectric materials have the potential to enhance triboelectric performances according to the relationship between the surface charge density and dielectric constant, the invention of triboelectric materials based on various polarization mechanisms enables the development of high-powered wearable devices, which can be achieved as follows:

1. Because a variety of high-*k* dielectric materials have been synthesized by controlling the structural factor [66] or chemical doping [67, 68], there are several candidates to increase the dielectric constant of polymer composites. Moreover, the surface modification of dielectric nanomaterials for homogeneous dispersion in the polymer matrix [69, 70] and the control of the dielectric structure (e.g., heterostructured multilayer composites [30, 31, 71, 72] or dielectric composites with aligned conductive materials [73, 74]) have been investigated to increase dielectric properties. However, few approaches have been utilized in triboelectric devices to enhance the output performance. The high compatibility or alignment of additives in the polymer matrix will enable an increase in the interfacial area or reduce the leakage current, which leads to the enhancement of the dielectric constant and the resultant output performance.
2. In addition to dielectric polymer nanocomposites, modifying polymer chain structures can enhance the dielectric properties because of the dipolar polarization through the improved dipole moments. Until now, polymeric materials with high dielectric constants have been synthesized by grafting polarizable components [58, 60] or by engineering nanostructures [61, 62, 75, 76], which increases the dielectric constant by dipolar polarization. Polymer-based dielectric materials are good candidates for use as triboelectric materials because of their physical properties, such as flexibility and solution-processability, which facilitate the development of printable triboelectric devices for next-generation wearable applications.
3. In addition to dielectric polarization, an electric poling process that can induce dipole realignment under a strong electric field can be another approach to improve the dielectric constant, which subsequently enables the enhancement of triboelectric performances [77–80]. Recently, self-poling methods have been applied to considerably improve ferroelectric properties via the shear-induced process [81] in piezoelectric generators, although the output performance remains lower than that of the triboelectric generators. The mechanism, combined with dielectric polarization and self-poling in dielectric composites, can be a synergistic effect to significantly improve the dielectric constant, leading to a remarkable enhancement of triboelectric performances.
4. Most studies have focused on negative triboelectric materials. Because triboelectric performance arises from the contact electrification between the positive and negative triboelectric layers, the positive triboelectric materials are an important factor toward enhancing output performances. Polarization-induced triboelectric pair materials can promote the development of triboelectric devices with significantly enhanced output performances, which facilitates practical applications requiring high-output power, such as smart wearable devices and portable IoT devices.

The article "High-Performance Triboelectric Devices via Dielectric Polarization: A Review" was published in 2021. Journal: Nanoscale Res Lett.

## Data Availability

Not applicable.

## Abbreviations

EDL: Electric double layer
PDMS: Polydimethylsiloxane
PET: Polyethylene terephthalate
PtBA: Poly(tert-butyl acrylate)
PTF: Poly(2,2,2-trifluoroethyl methacrylate)
PVA: Poly(vinyl alcohol)
PVDF: Polyvinylidene fluoride
SPE: Solid polymer electrolyte
